The article "The C2238/αANP Variant Is a Negative Modulator of Both Viability and Function of Coronary Artery Smooth Muscle Cells" was retracted in 2025. Reasons: errors in the data; errors in the images; duplicated images; overlap with earlier publications.

# The C2238/αANP Variant Is a Negative Modulator of Both Viability and Function of Coronary Artery Smooth Muscle Cells

**DOI:** 10.1371/journal.pone.0113108

**Published:** 2014-11-17

**Authors:** Speranza Rubattu, Simona Marchitti, Franca Bianchi, Sara Di Castro, Rosita Stanzione, Maria Cotugno, Cristina Bozzao, Sebastiano Sciarretta, Massimo Volpe

**Affiliations:** 1 IRCCS Neuromed, Pozzilli (Isernia), Italy; 2 Department of Clinical and Molecular Medicine, School of Medicine and Psychology, University Sapienza of Rome, Ospedale S. Andrea, Rome, Italy; The University of Tennessee Health Science Center, United States of America

## Abstract

**Background:**

Abnormalities of vascular smooth muscle cells (VSMCs) contribute to development of vascular disease. Atrial natriuretic peptide (ANP) exerts important effects on VSMCs. A common ANP molecular variant (T2238C/αANP) has recently emerged as a novel vascular risk factor.

**Objectives:**

We aimed at identifying effects of CC2238/αANP on viability, migration and motility in coronary artery SMCs, and the underlying signaling pathways.

**Methods and Results:**

Cells were exposed to either TT2238/αANP or CC2238/αANP. At the end of treatment, cell viability, migration and motility were evaluated, along with changes in oxidative stress pathway (ROS levels, NADPH and eNOS expression), on Akt phosphorylation and miR21 expression levels. CC2238/αANP reduced cell vitality, increased apoptosis and necrosis, increased oxidative stress levels, suppressed miR21 expression along with consistent changes of its molecular targets (PDCD4, PTEN, Bcl2) and of phosphorylated Akt levels. As a result of increased oxidative stress, CC2238/αANP markedly stimulated cell migration and increased cell contraction. NPR-C gene silencing with specific siRNAs restored cell viability, miR21 expression, and reduced oxidative stress induced by CC2238/αANP. The cAMP/PKA/CREB pathway, driven by NPR-C activation, significantly contributed to both miR21 and phosphoAkt reduction upon CC2238/αANP. miR21 overexpression by mimic-hsa-miR21 rescued the cellular damage dependent on CC2238/αANP.

**Conclusions:**

CC2238/αANP negatively modulates viability through NPR-C/cAMP/PKA/CREB/miR21 signaling pathway, and it augments oxidative stress leading to increased migratory and vasoconstrictor effects in coronary artery SMCs. These novel findings further support a damaging role of this common αANP variant on vessel wall and its potential contribution to acute coronary events.

## Introduction

Atrial natriuretic peptide (ANP) is a cardiovascular hormone which exerts several beneficial properties on both cardiovascular hemodynamic and structure [1]. Its vasorelaxant, diuretic and natriuretic effects are mediated by the membrane-bound guanylyl cyclase type A receptor (GC-A) through an increase of cyclic guanylate monophosphate (cGMP) levels. On the other hand, ANP binding to natriuretic peptide type C (NPR-C) receptor is known to mediate its clearance [1]. ANP exerts its vasodilatory property by inducing vascular smooth muscle cell (VSMC) relaxation [1]. Previous evidence indicates that ANP can also reduce VSMC proliferation [2]. Notably, microRNAs may be involved in these effects since miRNA-21 was shown to contribute to the antiproliferative effect of ANP in human aortic SMCs [3].

The article "The C2238/αANP Variant Is a Negative Modulator of Both Viability and Function of Coronary Artery Smooth Muscle Cells" was retracted in 2025. Reasons: errors in the data; errors in the images; duplicated images; overlap with earlier publications.

VSMCs play a relevant role in vessel physiology and disease [4]. In particular, based on their ability to adapt to various stimuli, they can participate to either the vascular repair process or to the vascular disease condition such as atherosclerotic plaque formation [5]. Importantly, VSMCs are also required to maintain stability of atherosclerotic plaques [6]. These evidences suggest that, by regulating VSMC biological functions, ANP may contribute to both physiological and pathological vascular processes.

The common T2238C molecular variant of human αANP is emerging as a novel cardiovascular risk factor for its ability to increase the risk of cardiovascular events both in coronary artery disease patients and in the general population [7]–[12], along with a significant impairment of endothelium-dependent vasodilation [13]. These negative effects result from deregulated activation of NPR-C by CC2238/αANP variant [13].

The impact of CC2238/αANP on VSMCs has not been explored yet. Since its understanding may integrate knowledge on mechanisms of vascular disease promotion dependent on this common αANP molecular variant, we performed the present studies to explore: 1) the effects of CC2238/αANP on coronary artery SMC (CASMC) viability, migration and motility; 2) the pathways underlying alterations of viability and function dependent on CC2238/αANP in CASMCs; 3) the implication of NPR-C driven cAMP/PKA/CREB pathway in modulating cellular viability through phosphoAkt and miR21 regulation in the presence of CC2238/αANP.

## Materials and Methods

### 1. Effects of exposure to TT2238 and CC2238/αANP in CASMCs

Commercially available CASMCs (human coronary artery smooth muscle cells obtained from normal donors, Cat. No CC-2583), purchased from Lonza (Walkersville, MD, USA), were grown in Smooth Muscle Growth Medium-2 (SmgM-2). They were used within the 5th passage and at 70% confluence for the following sets of experiments after an overnight exposure (12 hrs) to either TT2238/αANP (wild type) or CC2238/αANP (variant) at 10^−9^ M concentration, as previously reported for endothelial cells (ECs) [13]. This concentration has been used in our studies to better mimic the physiological condition of vascular cells exposed to both circulating and endogenous αANP. Once exposure to either αANP form was completed, variables described below were assessed 24 hrs later. From three to six experiments were performed for each of the following studies.

The article "The C2238/αANP Variant Is a Negative Modulator of Both Viability and Function of Coronary Artery Smooth Muscle Cells" was retracted in 2025. Reasons: errors in the data; errors in the images; duplicated images; overlap with earlier publications.

#### Cell viability assessment by trypan blue assay

Cells were seeded in 60-mm well plates (2×10^5^ cells/well), cultured in their medium for 24 hrs, and subsequently stimulated with either TT2238- or CC2238/αANP for 12 hrs in the presence of 10% fetal bovine serum (FBS). Twenty-four hrs later, viable and dead cells were counted using the Trypan blue exclusion method under an optical microscope, as previously described [13].

#### Cell viability assessment by Annexin V-PI staining

Counting of apoptotic cells was performed by flow cytometry analysis (FACS) using Annexin V-Fitc and Propidium Iodure (PI) staining (ImmunoStep, Salamanca, Spain). For this purpose, 24 hrs after completion of overnight exposure to either αANP form, CASMCs were harvested by incubation with 1 ml of trypsin/EDTA (Lonza) for 3 min at 37°C. Trypsinization was stopped by addition of medium and the suspension was centrifuged at 1200 rpm for 5 min. at 4°C. Each pellet was washed with cold phosphate buffered saline (PBS 1x). Then, tubes were vortexed thoroughly and centrifuged again as before. Cells were gently resuspended and vortexed in binding buffer at a concentration of 3×10^6^ cells/ml. Then, 100 µl of cell suspension was added to 5 µl of Annexin V-Fitc and 10 µl of PI. Samples were mixed for 15 min. in the dark at 4°C and 400 µl of PBS 1x was added to the solution. Ten thousand cells were analyzed by FACS on a BD Accuri C6 flow cytometer to count apoptotic cells. Both negative control (untreated cells) and positive control (cells treated with hydrogen peroxide) were included in the analysis.

#### Reactive oxygen species (ROS) levels assessment

Oxidative stress was evaluated 24 hrs after completion of exposure to either αANP form by applying the DCHF procedure, as previously described [13].

#### Cell migration assay

To test cell migration, CASMCs were seeded in 24-well plates (8×10^4^ cells/well), cultured in their medium for 24 hrs, subsequently starved and stimulated with either TT2238- or CC2238/αANP form for 12 hrs in the presence of 10% FCS. At the end of stimulation, cells were resuspended in their medium, starved and seeded in Boyden chambers (BD Biosciences, San Jose, California, USA) to test migration (chemotaxis). In fact, following a 24-hrs period of incubation, cells migrated from the upper part of the chamber to the lower filter were fixed by Diff Quick (Dade Behring, Paris, France) and visualized by microscopy. To test the involvement of both ROS and cAMP levels in modulating the migratory property of CASMCs upon CC2238/αANP, separate sets of experiments were perfomed in the presence of apocynin (200 mmol/l, Sigma) and of forskolin (FSK, 10 µM, Sigma).

The article "The C2238/αANP Variant Is a Negative Modulator of Both Viability and Function of Coronary Artery Smooth Muscle Cells" was retracted in 2025. Reasons: errors in the data; errors in the images; duplicated images; overlap with earlier publications.

#### Collagen gel lattice contraction assay

To test cell contraction, a commercially available kit assay was used (Cell Biolabs, San Diego, CA, USA). Two parts of cells were mixed with eight parts of collagen gel lattice mixture and they were plated for 1 hr at 37°C. Thereafter, 1 ml of medium was added and incubated for 2 days. Next, the gels were released from the sides of the wells and full release was allowed for 24 hrs. During the last 12 hrs of release either 10^−9^ M TT2238- or CC2238/αANP was added to cells. After completion of incubation, the area of gel lattice was taken with Image J software, and the relative lattice area was obtained by dividing the area of the well 24 hrs after detachment by the initial area of the well. To test the involvement of both ROS and cAMP levels in modulating cell motility upon CC2238/αANP, separate sets of experiments were performed in the presence of apocynin (200 mmol/l) and of FSK (10 µM).

### 2. Investigation of the signaling involved in the negative effects of CC2238/αANP in CASMCs

From three to six experiments were performed for each of the following studies, unless otherwise indicated.

#### Cyclic adenylate monophosphate (cAMP) and cyclic guanylate monophosphate (cGMP) levels measurement

For this purpose, CASMCs were seeded in six-well plates (2×10^5^ cells/well) and cultured in SmgM-2 medium for 24 hrs. At this time, they were first starved for 2 hrs and then pretreated for 30 min. with 0.1 mmol/L isobutylmethylxanthine (IBMX, Sigma) before stimulation with the conditioned medium containing IBMX 0.1 mM and either TT2238 or CC2238/αANP at 10^−9^ M concentration for 30 min., based on our own data [13] and on previously published protocols [14]. cGMP and cAMP measurements were performed with specific enzymeimmunoassay Biotrak (EIA) System (Amersham, Piscataway, New Jersey, USA), following the manufacturer’s instructions (number of experiments = 12). To better assess guanylyl cyclase activity following binding of both αANP forms with GC-A (natriuretic peptide type A receptor, NPR-A), a dose-response curve was performed by using a range of concentrations included between 10^−11^ and 10^−6^ M of each peptide. Furthermore, to support the involvement of NPR-C, rather than NPR-A, in mediating deleterious effects of CC2238/αANP, we assessed its impact on cell viability (by trypan blue) in the presence of 500 nM anantin (NPR-A antagonist that blocks cGMP release [15]).

The article "The C2238/αANP Variant Is a Negative Modulator of Both Viability and Function of Coronary Artery Smooth Muscle Cells" was retracted in 2025. Reasons: errors in the data; errors in the images; duplicated images; overlap with earlier publications.

#### Analysis of miR21 expression

At the end of exposure to either αANP form, microRNA from cells was immediately obtained using mirVana miRNA isolation kit (Applied Biosystems, CA, USA). The RT reaction for miR21 and for U75-control miR was performed using TaqMan MicroRNA Reverse Transcription Kit (Applied Biosystems, Milan, Italy). Two ng/µL of RNA, 1X stem-loop RT primer, 3.33 U/µL reverse transcriptase, 0.25 U/µL RNase inhibitor, 0.25 mM dNTPs, and 1X reaction buffer were run in a total reaction volume of 15 µL and incubated at 16°C for 30 min, 42°C for 30 min, and 85°C for 5 min in a thermal cycler. 0.8 µL of the RT reaction was combined with 0.5 µL of a specific TaqMan MicroRNA Assay (U75-control, miR-21, 20X; forward primer, reverse primer, and probe) and 5 µL of TaqMan Universal PCR Master Mix in a 10 µL final volume. Real-time (RT)-PCR was performed using an Applied Biosystems 7900HT Fast Real-Time PCR System with cycling conditions of 95°C for 10 min followed by 95°C for 15 sec and 60°C for 60 sec for a total of 40 cycles. Each TaqMan assay was run in triplicate. Results were expressed as relative levels of each microRNA comparing different treatments.

A separate set of studies tested the role of cGMP dependent kinase (cGK) in mediating the 50% miR21 reduction dependent on wild type αANP. We used cGK inhibitor (Rp-8-Br-PET-cGMPS, Sigma) at concentration of 25 µM for 30 min. followed by overnight exposure to wild type αANP.

#### Western blot analysis of Akt, NADPH (gp91 phox subunit), eNOS, miR21 targets (PDCD4, PTEN, Bcl2)

To determine protein expression levels 24 hrs after completion of exposure to either TT2238- or CC2238/αANP, samples were lysed in 1∶10 weight/volume in lysis buffer (50 mM NaCl, 100 mM Tris-HCl pH 7.4, 1 mM EDTA, 1% SDS) supplemented with protease and phosphatase inhibitors (Sigma). Samples were incubated on ice for 15 min. and centrifuged at 13000 rpm for 15 min. Protein concentration was determined by DC Protein Assay Kit (Bio-Rad, Hercules, CA, USA) following manufacturer’s instructions. Protein lysates were boiled at 95°C for 10 min. in presence of gel loading buffer (Bio-Rad). 50 µg of each sample were loaded on 10% SDS-polyacrylamide gel and run for 120 min. at 100 V. Proteins were then transferred to polyvinylidene difluoride membranes (Amersham) using the Trans-Blot Turbo Transfer System (Bio-Rad). Non specific binding sites were blocked at room temperature for 1 hr in 5% skim-milk in Tris-buffered saline buffer +0.1% Tween 20 (Sigma) (TBS-T). Membranes were incubated at 4°C overnight with primary antibodies diluted in 5% bovine serum albumine (BSA) in TBS-T. The following primary antibodies were used: 1∶200 rabbit polyclonal anti-protein kinase B (Akt) (Cat. No. 9272) and 1∶200 rabbit polyclonal anti-p-Akt (Ser413) (Cat. No. 9271) both purchased from Cell Signaling Technologies (Danvers, MA, USA); 1∶200 donkey polyclonal antibody anti-gp91-phox subunit of nicotinamide adenine dinucleotide phosphate (NADPH) (Cat. No. sc-5827, Santa Cruz Biotechnology, Santa Cruz, CA, USA); 1∶200 mouse monoclonal anti-endothelial nitric oxide synthase (eNOS), Cat. No 5880, Cell Signaling; 1∶200 rabbit polyclonal antibody anti-phospho-eNOS (Ser1177) Cat. No 9571, Cell Signaling; 1∶200 rabbit monoclonal antibody anti-phosphatase and tensin homolog (PTEN) (Cat. No 9559, Cell Signaling); 1∶200 rabbit monoclonal anti-programmed cell death protein 4 (PDCD4), Cat. No 9535, Cell Signaling; 1∶200 rabbit polyclonal anti-B-cell lymphoma 2 (Bcl2), Cat. No sc-492, Santa Cruz Biotechnology; 1∶5000 anti-β-actin (Cat. No A5441, Sigma) used as housekeeping gene. Following three washes of 10 min. in TBS-T, membranes were incubated for 1 hr at room temperature with 1∶5000 horseradish peroxidase-conjugated secondary antibody goat anti-rabbit (Cat. No sc-2004, Santa Cruz) or goat anti-mouse (Cat. No sc-2005, Santa Cruz) diluted in 5% BSA. After three washes of 10 min. in TBS-T, signals were revealed with an enhanced chemiluminescence detection system (Luminata Crescendo, Millipore, Darmstadt, Germany) and the immunoreactivity of bands was visualized on a high-performance chemiluminescence apparatus (ChemiDoc MP System, Bio-Rad). Protein bands were scanned and quantified densitometrically. They were finally normalized using β-actin levels.

The article "The C2238/αANP Variant Is a Negative Modulator of Both Viability and Function of Coronary Artery Smooth Muscle Cells" was retracted in 2025. Reasons: errors in the data; errors in the images; duplicated images; overlap with earlier publications.

### 3. Impact of NPR-C gene silencing in CASMCs in the presence of CC2238/αANP

NPR-C gene silencing was performed once cells had reached 70% confluence. At this time, they were washed with PBS 1x, and OPTI-MEM-reduced serum medium (Invitrogen, Milan, Italy) was added to the cells. Two NPR-C specific small interfering RNAs (Mission siRNA, Sigma) and a nucleic acid transferring agent (RNA I Max lipofectamine, Invitrogen) were incubated in OPTI-MEM reduced serum medium for 20 min. at room temperature to form a siRNA-lipofectamine complex. The siRNA-lipofectamine complex-containing medium was added to the cells to a final siRNA concentration of 50 nM. Five hrs later, the complex-containing medium was replaced with SmgM-2 supplemented with 10% FBS. Cells transfected with lipofectamine and nonsense siRNA (Sigma Aldrich) were used as control. Twenty-four hrs later, both silenced and not silenced cells were exposed to CC2238/αANP for 12 hrs and subsequently analyzed for: cell viability, eNOS and NADPH protein expression levels, ROS levels, cell migration, cell contraction, miR21 and related targets (PTEN, PDCD4, Bcl2) expression, Akt phosphorylation levels. Six experiments were performed for these studies.

The article "The C2238/αANP Variant Is a Negative Modulator of Both Viability and Function of Coronary Artery Smooth Muscle Cells" was retracted in 2025. Reasons: errors in the data; errors in the images; duplicated images; overlap with earlier publications.

### 4. Impact of miR21 overexpression in CASMCs in the presence of CC2238/αANP

Cells were used at 70% confluence. Mimic hsa-miR21 (Mission microRNA, Sigma) and RNA I Max lipofectamine were incubated in OPTI-MEM reduced serum for 20 min. at room temperature to form a mimic-lipofectamine complex. The complex containing medium was added to the cells to reach a final mimic miR21 concentration of 100 nM. Five hrs later the complex containing medium was replaced with SmGM-2 supplemented with 10% FBS. Cells transfected with lipofectamine and Mission miRNA negative control (Sigma) were used as control. Twenty-four hrs after transfection cells overexpressing miR21 were exposed to CC2238/αANP for 12 hrs and used, 24 hrs later, for evaluation of: cell viability, ROS levels, NADPH and eNOS expression, cell migration and cell contraction, modulation of miR21 molecular targets (PTEN, PDCD4, Bcl2) and of Akt phosphorylation. Efficacy of miR21 overexpression was verified by RT-PCR, as reported above, at both two and four days following transfection. Six experiments were performed for these studies.

### 5. Is the NPR-C driven cAMP/Protein kinase A (PKA)/CREB axis related to miR21 and pAkt regulation in CASMCs upon CC2238/αANP exposure?

To explore the role of cAMP/PKA/CREB axis in CC2238/αANP dependent effects on CASMC viability, we evaluated both miR21 and Akt phosphorylation expression in the following sets of experiments:

-CC2238/αANP was co-incubated with 10 µM FSK (in order to increase intracellular cAMP levels), as previously reported [13]. At the end of stimulation, we assessed expression levels of miR21 and, 24 hrs later, of Akt phosphorylation (as described above).
-CC2238/αANP was co-incubated with 10 µM FSK and 15 µM Dihydrochloride hydrate (H89, PKA inhibitor, Sigma). Modulation of both miR21 expression and pAkt phosphorylation levels was assessed as specified above.
-CC2238/αANP was co-incubated with 10 µM FSK following either 60 or 120 min. pre-incubation with 25 µM p300/CREB(CBP) (CREB inhibitor, Sigma). Modulation of both miR21 expression and pAkt phosphorylation levels was assessed as specified above.

### Statistical Analysis

Continuous variables are expressed as mean±SEM. Comparisons between 2 groups were performed using Student t test. When the analysis was adjusted for the multiplicity of compared groups, 1-way ANOVA followed by Bonferroni post hoc test was performed. SPSS statistical software (SPSS Inc, Chicago, IL, version 12.0) was used for statistical analysis.

The article "The C2238/αANP Variant Is a Negative Modulator of Both Viability and Function of Coronary Artery Smooth Muscle Cells" was retracted in 2025. Reasons: errors in the data; errors in the images; duplicated images; overlap with earlier publications.

A p<0.05 was considered significant.

## Results

### Effects of exposure of TT2238- and CC2238/αANP on cell viability, oxidative stress, migration and contraction in CASMCs

Cell viability was significantly impaired in cells exposed to CC2238/αANP (Fig. 1A, 1B, S1A). Consistently, apoptosis and necrosis were significantly increased by variant αANP (Fig. 1B, S1A). ROS levels were also markedly increased (Fig. 1C), along with a significant increase of gp91-phox subunit of NADPH expression and a significant decrease of phosphorylated eNOS expression (Fig. 1D).

**Figure 1:** Effects of exposure to either TT2238- or CC2238/αANP on viability and oxidative stress in CASMCs. A. Cell vitality as determined by trypan blue (n = 4); B. Cell vitality as assessed by FACS (n = 4): representative scatter plots are shown with percentages of live cells (bottom left), early apoptotic cells (upper left), late apoptotic cells (upper right), necrotic cells (bottom right); C. ROS levels (n = 6); D. NADPH and eNOS expression levels (n = 3). Representative western blots are shown; bars represent results of densitometric analysis. Control (CTR): untreated cells; positive control: cells treated with H_2_O_2_.♦p<0.01; for all other comparisons p<0.0001.

CC2238/αANP induced a marked increase of cell migration, as compared to TT2238/αANP (Fig. 2A), consistently with previous observations obtained in ECs [16]. A significant increase of cell contraction was detected upon CC2238/αANP exposure (Fig. 2B).

**Figure 2:** Effects of exposure to either TT2238- or CC2238/αANP on cell migration and cell contraction. Photos of cell migration (A) and of cell contraction (B) upon exposure of CASMCs to either TT2238/αANP or CC2238/αANP as compared to control (CTR). Results are plotted in the graphs at the bottom of the figure. Number of experiments = 4. *#p<0.0001.

### Investigation of the signaling involved in the negative effects of CC2238 vs TT2238/αANP in CASMCs

Release of cAMP levels was dramatically reduced by CC2238/αANP, in contrast to wild type αANP (Fig. 3A). Levels of cGMP were remarkably increased by both wild type and variant αANP at all tested concentrations (Fig. 3B, S2A). Blocking of NPR-A with anantin did not avoid the deleterious effects of CC2238/αANP on cell viability, and it was associated with a marked cAMP levels decrease (S2B). Degree of Akt phosphorylation was significantly reduced by αANP variant only, similarly to what has been previously reported in ECs [13] (Fig. 3C).

**Figure 3:** Investigation of the signaling involved in the negative effects of CC2238/αANP in CASMCs. cAMP (A) and cGMP (B) levels (number of experiments = 12) (for all comparisons p<0.0001); C. pAkt/Akt levels with representative western blot and results of densitometric analysis (n = 4); D. hsa-miR21 expression levels as determined by RT-PCR (n = 6) (for all comparisons p<0.0001); E. miR21 molecular targets expression levels under either TT2238/αANP or CC22338/αANP exposure (n = 3). Representative western blots are shown; bars represent results of densitometric analysis. (♦p<0.01; for all other comparisons p<0.0001). CTR = control.

The article "The C2238/αANP Variant Is a Negative Modulator of Both Viability and Function of Coronary Artery Smooth Muscle Cells" was retracted in 2025. Reasons: errors in the data; errors in the images; duplicated images; overlap with earlier publications.

Based on previous findings showing involvement of miR21 downregulation in the anti-proliferative effect of wild type αANP in aortic SMCs [3], we compared degree of miR21 modulation under either TT2238- or CC2238/αANP exposure. A marked suppression of miR21 expression was revealed upon exposure to CC2238/αANP, whereas TT2238/αANP reduced miR21 expression by 50% (Fig. 3D). Notably, the TT2238/αANP effect on miR21 was mediated by cGMP dependent kinase (S3), confirming previous data [3].

Known targets of miR21 are Bcl2, PTEN and PDCD4 that are all involved in cell apoptosis, proliferation and growth (17–19). In fact, as a consequence of miR21 suppression, CC2238/αANP reduced Bcl2 expression and significantly increased both PTEN and PDCD4 expression levels (Fig. 3E), as key mechanisms underpinning its deleterious effects.

### Impact of NPRC gene silencing on detrimental effects induced by CC2238/αANP

Silencing of NPR-C gene abolished the effects induced by CC2238/αANP on cell viability, cell apoptosis and necrosis (S1B). It also blunted ROS levels accumulation induced by CC2238/αANP (Fig. 4A). Both Akt phosphorylation (Fig. 4B) and miR21 expression (Fig. 4C) were restored. Consequent changes of expression of miR21 related targets (PDCD4, Bcl2, PTEN) are shown in S4 (panels A–C). In addition, NADPH and eNOS protein expression were both rescued (S4, panels D, E). Both increased migration and increased contraction dependent on CC2238/αANP were abolished (S5).

**Figure 4:** Impact of NPR-C gene silencing on detrimental effects induced by CC2238/αANP in CASMCs. A. ROS levels (n = 6); B. pAkt/Akt levels with representative western blot and results of densitometric analysis (n = 3); C. miR21 expression levels in NPR-C gene silenced cells upon exposure to CC22338/αANP (n = 6). Control (CTR): untreated cells; positive control: cells treated with H_2_O_2_. siRNA1 and siRNA2 = small interfering RNAs for NPR-C gene silencing. For all comparisons p<0.0001.

### Impact of miR21 overexpression in the presence of CC2238/αANP

In order to test whether the dramatic reduction of miR21 expression levels is involved in the detrimental effects induced by CC2238/αANP in CASMCs, we overexpressed miR21 in cells exposed to variant αANP. Overexpression of miR21 was confirmed by RT-PCR (S6). Concomitant overexpression of miR21 with exposure to CC2238/αANP restored cell viability, reduced cell apoptosis and necrosis (Fig. S1C), reduced ROS levels (Fig. 5A), rescued phosphorylated Akt levels (Fig. 5B), increased eNOS and reduced NADPH expression (Fig. 5C, 5D). In this experimental condition, Bcl2 expression increased whereas both PTEN and PDCD4 expression decreased as expected (Fig. 6). Overexpression of miR21 reduced cell migration stimulated by CC2238/αANP, whereas it was unable to counteract the degree of cell contraction dependent on CC2238/αANP (S7).

The article "The C2238/αANP Variant Is a Negative Modulator of Both Viability and Function of Coronary Artery Smooth Muscle Cells" was retracted in 2025. Reasons: errors in the data; errors in the images; duplicated images; overlap with earlier publications.

**Figure 5:** Impact of miR21 overexpression in CASMCs in the presence of CC2238/αANP. A. ROS levels (n = 6); B. pAkt/Akt levels with representative western blot and results of densitometric analysis (n = 3); eNOS (C) and NADPH (D) expression levels with representative western blot and results of densitometric analysis in cells overexpressing miR21 and concomitantly exposed to CC22338/αANP (n = 3). Control (CTR): untreated cells; positive control: cells treated with H_2_O_2_. For all comparisons p<0.0001.

**Figure 6:** miR21 targets expression levels under miR21 overexpression and concomitant exposure of CASMCs to CC2238/αANP. Representative western blots are shown; bars represent results of densitometric analysis. Number of experiments = 4. For all comparisons p<0.0001. CTR = control.

Of note, miR21 overexpression alone was able to induce the expected changes on its own targets and on phosphoAkt levels (Fig. 5B, Fig. 6). Furthermore, the known stimulating effect on VSMC contraction [3] was confirmed (S7).

### ROS levels directly influence CASMC migration and contraction upon CC2238/αANP exposure

As shown in S8, apocynin abolished the stimulation of both migration and contraction upon exposure to CC2238/αANP. The contribution of increased cAMP levels to migration and contraction (tested in the presence of FSK) was comparable to that of increased oxidative stress.

### cAMP/PKA/CREB axis modulates miR21 and phosphoAkt expression levels upon CC2238/αANP in CASMCs

Co-incubation of CC2238/αANP with FSK allowed a significant increase of both miR21 and phosphoAkt expression levels, as compared to cells treated with CC2238/αANP only (Fig. 7A, 7B, 7C). In the presence of concomitant exposure to CC2238/αANP, FSK and H89 both miR21 and phosphoAkt levels were unable to increase as much as in the presence of FSK only (Fig. 7). The same results were obtained when cells were exposed to CC2238/αANP, FSK and CREB inhibitor (Fig. 7). These data demonstrate that inhibition of cAMP/PKA/CREB axis does not allow the recovery of both miR21 and phosphoAkt expression levels in the presence of CC2238/αANP.

The article "The C2238/αANP Variant Is a Negative Modulator of Both Viability and Function of Coronary Artery Smooth Muscle Cells" was retracted in 2025. Reasons: errors in the data; errors in the images; duplicated images; overlap with earlier publications.

**Figure 7:** Evidence that cAMP/PKA/CREB axis regulates miR21 expression and Akt phosphorylation in CASMCs. A. miR21 expression levels upon concomitant exposure of CASMCs to: CC2238/αANP and FSK; CC2238/αANP, FSK and H89; CC2238/αANP, FSK and CREB inhibitor p300/CREB(CBP); the latter was pre-incubated either 60 or 120 min. followed by exposure to CC2238/αANP and FSK; B and C. pAkt/Akt expression levels in the same experimental conditions. Number of experiments = 6. For all comparisons p<0.0001.

## Discussion

The present study explored the impact of CC2238/αANP in VSMCs, a fundamental cellular element for vessel wall physiology and disease, and it demonstrated for the first time that CC2238/αANP is a highly deleterious factor for coronary artery SMCs, as compared to wild type αANP.

The main original findings of the current set of data can be summarized as follows: 1) identification of a strong contribution of miR21 suppression in mediating the deleterious effects on CASMC viability exerted by CC2238/αANP; 2) first demonstration that NPR-C/cAMP/PKA/CREB axis is involved in modulation of both miR21 and Akt phosphorylation in CASMCs upon CC2238/αANP; 3) first evidence that CC2238/αANP is a significant promoter of both CASMC migration and contraction, mainly dependent on ROS accumulation, and therefore it exerts vascular functional properties different from those of regular αANP (S9).

ANP is involved in the control of cardiac and vascular remodeling by performing anti-proliferative effects on cardiac, endothelial and SM cells [1], [2], [20]. Functional derangements due to either circulating peptide levels or peptide structure lead to pathological states within the cardiovascular system [21].

The common T2238C/αANP molecular variant has recently emerged as a novel cardiovascular risk factor for its ability to alter the physiological beneficial properties of regular αANP. Apart from the previously identified effects on EC viability and function [13], [16], we now demonstrate its deleterious actions in VSMCs.

The effects of CC2238/αANP in CASMCs were mediated by NPR-C activation, similarly to what has been first discovered in ECs, and strictly dependent on the higher affinity binding of CC2238/αANP with NPR-C [13]. In fact, CC2238/αANP led to a significant reduction of CASMC viability and of cAMP levels, dependent on NPR-C driven adenylate cyclase inhibition, even when NPR-A was blocked by the use of anantin. Consistently, NPR-C gene silencing abolished all effects due to αANP variant. Of note, the functional consequences of pathological activation of NPR-C by CC2238/αANP strongly differ from those obtained through physiological stimulation with its agonist, i.e. CNP, mainly consisting in beneficial effects on vascular cells [22].

The article "The C2238/αANP Variant Is a Negative Modulator of Both Viability and Function of Coronary Artery Smooth Muscle Cells" was retracted in 2025. Reasons: errors in the data; errors in the images; duplicated images; overlap with earlier publications.

The microRNA-21, that is strongly involved in the effects dependent on CC2238/αANP in CASMCs, is emerging as a fundamental protective factor for maintaining vitality and proliferation in several cell types and it has been found to be highly expressed in all main types of cardiovascular cells [23]. It plays important roles in VSMC proliferation and apoptosis through the targeting of PTEN, Bcl2 and PDCD4 proteins [17]–[19]. The known anti-proliferative effect of wild type αANP has been previously shown to associate with a decrease of miR21 in aortic SMCs, whereas overexpression of miR21 restored VSMC proliferation [3]. In our experimental setting, we observed that miR21 levels were completely suppressed by CC2238/αANP as compared to wild type αANP (that caused 50% reduction). Accordingly, expression levels of miR21 molecular targets were remarkably changed by αANP variant. The miR-21 suppression appeared to be tightly related to all negative effects observed upon CC2238/αANP. In fact, overexpression of miR21 rescued expression levels of its molecular targets and of Akt phosphorylation, while restoring cell viability. Our results imply that suppression of miR21 upon CC2238/αANP contributes to cause detrimental effects in VSMCs, whereas reduction of miR21, mediated by cGMP dependent kinase, produces the physiological anti-proliferative effect of wild type αANP.

Notably, we support evidence that miR21 belongs to Akt regulatory network in cardiovascular cells, as an upstream factor, due to its ability to inhibit PTEN and to exert, through consequent increased Akt activity, important effects on cell proliferation [17], [24]. In fact, both PTEN and Akt represent key molecules for cell growth and survival, as well as for development of many cardiovascular diseases [25]–[27]. In our experimental context, miR21 suppression, dependent on CC2238/αANP, led to PTEN upregulation. In turn, miR21 overexpression reduced PTEN and, in the presence of CC2238/αANP, prevented the increase of PTEN expression. Finally, Akt phosphorylation was modulated in a manner consistent with PTEN changes.

Current knowledge on receptors involved in miRNA expression modulation is scarce. Activation of NPR-A has been suggested as the responsible mechanism for modulation of several miRNAs, including miR21, by wild type αANP in aortic SMCs [3]. We provide original evidence that deregulated activation of NPR-C, upon exposure to variant αANP, suppresses expression levels of miR21 in CASMCs. In fact, cells exposed to CC2238/αANP, in the absence of NPR-C, showed regular expression levels of miR21.

The article "The C2238/αANP Variant Is a Negative Modulator of Both Viability and Function of Coronary Artery Smooth Muscle Cells" was retracted in 2025. Reasons: errors in the data; errors in the images; duplicated images; overlap with earlier publications.

Previous studies have shown the ability of cAMP/PKA to regulate expression levels of few miRNAs, such as miR1 [28], miR335 [29], and miR375 [30]. Herein, we report the first evidence that cAMP/PKA/CREB pathway modulates miR21 expression in CASMCs. In fact, PKA inhibition by H89 did not allow the recovery of miR21 levels in the presence of FSK, upon stimulation with CC2238/αANP. Inhibition of CREB, cAMP responsive element, by p300/CREB(CBP) led to identical results. Thus, we support knowledge on the ability of cAMP/PKA/CREB axis to regulate expression of miRNAs in vascular cells.

Migration and contraction are fundamental processes for vascular remodeling, proliferation and disease [31], [32]. Herein, we show that CC2238/αANP is a strong promoter of CASMC migration and contraction, mainly dependent on ROS accumulation. In fact, decreases of ROS levels prevented both migration and contraction in the presence of αANP variant. The strong contribution of ROS to vascular cell migration and contraction are known [33], [34].

It is also worthwhile observing that miR21, when overexpressed in the presence of αANP variant, antagonized the effect of the latter with regard to migration but it was unable to antagonize the contractile property of CC2238/αANP. This evidence is consistent with the notion that miR21 exerts VSMC contraction through an independent activation of DOCK proteins [35].

Notably, CC2238/αANP exerted CASMC contraction despite miR21 suppression. The demonstration of a significantly increased vasoconstriction dependent on CC2238/αANP, in contrast to the known vasodilation promoted by wild type αANP, represents an important achievement of the current study. An increased vasoconstriction, along with the previously reported endothelial-dependent impaired vasorelaxation [13], constitutes a rational pathological substrate for higher predisposition to plaque instability and for an augmented rate of acute coronary and cerebrovascular events observed in CC2238/αANP carriers, as documented by several in vivo studies [7]–[12]. The recent demonstration that VSMCs stabilize atherosclerotic plaques [6] and that VSMC death and reduced proliferation promote plaque instability [36] further support our conclusions on the potential mechanisms, involving VSMCs, underpinning increased rate of acute cardiovascular events in CC2238/αANP carriers.

Few limitations of the study need to be acknowledged. We were unable to reproduce in vitro, for obvious technical limitations, the effects of the CT heterozygous peptide. On the other hand, it is assumed that heterozygous subjects carry 50% of both αANP forms.

The article "The C2238/αANP Variant Is a Negative Modulator of Both Viability and Function of Coronary Artery Smooth Muscle Cells" was retracted in 2025. Reasons: errors in the data; errors in the images; duplicated images; overlap with earlier publications.

In addition, although the current in vitro data were obtained in a cell line relevant for the human disease, we cannot extend them to other vascular beds. Finally, the in vivo implications of our findings remain to be assessed.

In conclusions, based on the current results, CC2238/αANP exerts deleterious effects on viability and function of CASMCs and it does it through binding with NPR-C, involvement of cAMP/PKA/CREB/miR21 pathway and marked increase of oxidative stress. The reduced proliferation and increased contraction of CASMCs may contribute to explain the augmented rate of acute coronary events in CC2238/αANP carriers. Pharmacological targeting of molecular pathways activated by CC2238/αANP may be proposed as a valuable strategy to reduce cardiovascular risk in subjects bearing this αANP variant.

## Supporting Information

Figure S1 **Graphical representation of FACS analysis in the different experimental settings.** Bars represent counts of live cells, early and late apoptotic cells, necrotic cells upon exposure of CASMCs to CC2238/αANP alone (A), in the presence of NPR-C gene silencing (B), and in the presence of miR21 overexpression (C). siRNA1 and siRNA2 = small interfering RNAs for NPR-C gene silencing. Number of experiments = 4. For all comparisons of CC2238/αANP vs other treatments: p<0.0001.
(TIF)

Figure S2 **A. cGMP levels in response to different concentrations of both TT2238- and CC2238/αANP (number of experiments = 5); B. Left panel = CASMC vitality as assessed by trypan blue upon CC2238/αANP exposure in the presence of anantin; levels of cGMP (middle panel) and of cAMP (right panel) upon CC2238/αANP exposure in the presence of anantin (number of experiments = 4); For all comparisons: p<0.05.**
(TIF)

Figure S3 **miR21 expression levels upon TT2238/αANP either in the absence or in the presence of cGK inhibitor.** Number of experiments = 3. For all comparisons: p<0.05.
(TIF)

Figure S4 **Impact of NPR-C gene silencing on protein expression levels upon concomitant exposure to CC2238/αANP.** miR21 targets expression levels (A, B, C); NADPH (D) and eNOS (E) expression levels. Representative western blots are shown; bars represent results of densitometric analysis. Number of experiments = 4. For all comparisons p<0.0001. CTR = control.
(TIF)

Figure S5 **Impact of NPR-C gene silencing on cell migration and cell contraction upon concomitant exposure to CC2238/αANP.** Photos of cell migration (A) and of cell contraction (B) under NPR-C gene silencing in the presence of CC2238/αANP. Results are plotted in the graphs at the bottom of the figure. siRNA1 and siRNA2 = small interfering RNAs for NPR-C gene silencing. Number of experiments = 6. For all comparisons p<0.0001.
(TIF)

Figure S6 **Overexpression of miR21 in CASMCs confirmed by RT-PCR.** Overexpression was verified at both 2 (A) and 4 (B) days following transfection. Number of experiments = 3.
(TIF)

Figure S7 **Impact of miR21 overexpression on cell migration and cell contraction upon concomitant exposure to CC2238/αANP.** Photos of cell migration (A) and of cell contraction (B) under miR21 overexpression and concomitant exposure to CC2238/αANP. Results are plotted in the graphs at the bottom of the figure. Number of experiments = 7. For all comparisons p<0.0001.
(TIF)

Figure S8 **Impact of co-incubation of CC2238/αANP with apocynin and FSK on both cell migration and cell contraction.** Photos of cell migration (A) and of cell contraction (B) upon exposure of CASMCs to CC2238/αANP with or without apocynin and FSK. Results are plotted in the graphs at the bottom of the figure. Number of experiments = 5. FSK = forskolin. For all comparisons p<0.0001.
(TIF)

Figure S9 **Schematic representation of the proposed pathways underlying the deleterious effects on cell viability and function exerted by CC2238/αANP in CASMCs through pathological involvement of NPR-C.**
(TIF)
